# A Methylene Blue Assisted Electrochemical Sensor for Determination of Drug Resistance of *Escherichia coli*

This article has been retracted.

**DOI:** 10.3389/fchem.2021.689735

**Published:** 2021-05-31

**Authors:** Rongshuai Duan, Xiao Fang, Dongliang Wang

**Affiliations:** ^1^ Department of Food and Drugs, Shandong Institute of Commerce and Technology, Jinan, China; ^2^ Qilu Medical University, Jinan, China; ^3^ Dong-E E-Jiao Co. Ltd., Liaocheng, China

**Keywords:** graphene, drug resistant, *Escherichia coli*, glassy carbon electrode, methylene blue

## Abstract

Due to the abuse of antibiotics in clinical, animal husbandry, and aquaculture, drug-resistant pathogens are produced, which poses a great threat to human and the public health. At present, a rapid and effective drug sensitivity test method is urgently needed to effectively control the spread of drug-resistant bacteria. Using methylene blue as a redox probe, the electrochemical signals of methylene blue in drug-resistant *Escherichia coli* strains were analyzed by a CV method. Graphene ink has been used for enhancing the electrochemical signal. Compared with the results of the traditional drug sensitivity test, we proposed a rapid electrochemical drug sensitivity test method which can effectively identify the drug sensitivity of *Escherichia coli*. The sensitivity of four *E. coli* isolates to ciprofloxacin, gentamicin, and ampicillin was tested by an electrochemical drug sensitivity test. The respiratory activity value %RA was used as an indicator of bacterial resistance by electrochemical method.

## Introduction

*Escherichia coli* is a Gram-negative short bacillus, and it is also the most important and the most abundant bacteria in the intestines of human beings and many animals (Jijie et al., 2018; Thakur et al., 2018). For a long time, it was thought that *E. coli* was not pathogenic in general, but some *E. coli* with special serotypes were found to be pathogenic to humans and animals, causing diarrhea, adult pleurisy, and septicemia. Food safety is one of the most important food safety problems (Brosel-Oliu et al., 2018; Zhou et al., 2018). With the abuse of antibiotics in clinic, animal husbandry, and aquaculture, the problem of antibiotic resistance of bacteria in the world is becoming increasingly serious. Foodborne drug-resistant bacteria may transmit drug resistance and drug-resistant genes to humans through food chain, thus causing human infection (Gomez-Cruz et al., 2018; Zhu et al., 2018). As an important mediator of drug-resistant genes, *E. coli* has the characteristics of easily producing drug resistance and a rapid variation of drug resistance. Its resistance spectrum will be further expanded with the change of time, which undoubtedly increases the harm of *E. coli*. In order to control the food safety problems caused by foodborne pathogens from the source, effective drug sensitivity detection methods are of great significance to prevent and control the infection and spread of foodborne drug-resistant bacteria (Hua et al., 2018; Yao et al., 2018; Zeinhom et al., 2018).

In recent years, electrochemical methods have been reported in the ultrasensitive detection of bacteria (Zheng et al., 2019; Karimi-Maleh et al., 2020a, 2021a). The principle of electrochemical detection of bacterial drug sensitivity is mainly based on the electron transfer of respiratory chain in bacterial energy metabolism (Fu et al., 2019; Xu et al., 2020; Zhang et al., 2020; Zhou et al., 2020; Nodehi et al., 2021a; Nodehi et al., 2021b). The respiration of bacteria involves the directional and orderly transfer of electroactive particles and the redox reaction of cellular substances (Khodadadi et al., 2019; Shamsadin-Azad et al., 2019; Karimi-Maleh et al., 2020b). The electrochemical changes of respiratory chain activity can be detected by electrochemical methods. The respiratory activity of bacteria can be observed by analyzing the electrical signals of redox probes so as to determine the drug sensitivity of bacteria. Ertl et al. (2000) and Ertl et al. (2003) used potassium ferricyanide as redox probe to explore an electrochemical method for the detection of drug sensitivity of *E. coli*. They treated *E. coli* with antibiotics for 20 min and then measured the electrical signals in the solution containing potassium ferricyanide to determine the drug sensitivity of the bacteria. The results were consistent with the traditional paper diffusion method. This method can provide a report within 25 min, but the IC_50_ value of penicillin and chloramphenicol is 100 times higher than that of the standard method. Chotinantakul et al. (2014) improved the experimental scheme. After the interaction between *E. coli* and bacteria, antibiotics were removed by centrifugation and then added to the test solution containing potassium ferricyanide to eliminate the influence of antibiotics on electrochemical test. This method can give the results of drug sensitivity test in 36 h.

With the development of microcomputer processing technology, the size of electrode can be reduced to micron or even nano level, which provides a technical support for the development of portable rapid detection system for drug-resistant bacteria (Naderi Asrami et al., 2020; Baghayeri et al., 2021; Karimi-Maleh et al., 2021b; Karimi-Maleh et al., 2021c). Besant et al. Besant et al. (2015) limited the volume of bacterial solution in a container of 2.75 nL and detected the reduction of azurol by electrochemical method to reflect the bacterial metabolic activity. This rapid electrochemical drug sensitivity test method can report the drug sensitivity of bacteria within 1 h.

Methylene blue (MB) is a dye widely studied in photodynamics. At the same time, due to its electrochemical characteristics, there are also some studies on its application in the field of chemically modified electrodes (Cui et al., 2018; Guo et al., 2018; Yao et al., 2018; Taghdisi et al., 2019). The blue MB can be reduced to colorless l mb by bacterial respiration, and the greater the bacterial count, the shorter the fading time of methylene blue. Due to its redox properties, MB is often used as a redox probe in electrochemical detection (Yu et al., 2019). Graphene has been frequently used for surface modification of electrochemical sensors since its discovery. Its excellent electrical properties can greatly enhance the sensing signal. Based on the theory of electron transfer in the process of energy metabolism of bacteria, the electrochemical characteristics of MB in *E. coli* from food sources *in vivo* were studied by using MB as a redox probe. Graphene ink has been used for electrode surface modification. Combined with traditional drug sensitivity test methods, we constructed a fast, sensitive, portable, and low-cost electrochemical sensor system for a rapid detection of drug resistance of foodborne bacteria.

## Materials and Methods

Reagents: methylene blue, potassium dihydrogen phosphate, potassium hydrogen phosphate, trisodium citrate, magnesium sulfate, calcium chloride, ammonium sulfate, ammonium chloride, and ammonium formate were purchased from Aladdin Co., Ltd. Graphene ink was purchased from Lowye Tech. Co., Ltd. Tryptone, agar powder, and yeast extract powder were purchased from Tianchen Biological Reagent Co., Ltd. Ciprofloxacin, gentamicin, and ampicillin were purchased from Shanghai Yeyuan Biotech. Co., Ltd. *E. coli* ATCC25922 was purchased from Guangdong Huankai Co., Ltd. All-field *E. coli* (E1–E4) were collected from Qilu Medical University. Table 1 shows the antibiotic susceptibility test results of E1–E4 toward ciprofloxacin, gentamicin, and ampicillin.

**TABLE 1:** Antibiotic susceptibility test results of E1–E4 toward ciprofloxacin, gentamicin, and ampicillin.

Strain	Antibiotics		
	**Ciprofloxacin**	**Gentamicin**	**Ampicillin**
E1	S	S	R
E2	R	S	R
E3	R	R	R
E4	R	R	S

LB broth: weigh 20 g tryptone, 20 g sodium chloride, and 10 g yeast extract, respectively, heat them, and dissolve them in 2,000 ml pure water. After adjusting pH to 7.2, the mixture was poured into conical flasks at 120°C. The mixture was sterilized with high-pressure steam for 15 min and then cooled them for standby.

LB agar: weigh 20 g tryptone, 20 g sodium chloride, 10 g yeast extract, and 30 g agar powder and heat them into 20,00 ml pure water. Adjust the pH to 7.2 and transfer into conical flasks, sterilize with 120°C high-pressure steam for 15 min, and then keep them in a 60°C water bath.

Colony count of *E. coli* ATCC 25922: The LB agar at 60 °C was poured into the culture dish. The agar in each culture dish was about 5 mm high. After the bacterial solution was diluted with 10 times of normal saline, three samples with appropriate dilution were selected, and 100 μL homogenate was added into the plate for coating. At the same time, take 100 μL blank diluent and add two sterile plates as blank control. The plate was inverted and cultured in 37 °C incubator for 24 h, and the colony count was conducted.

Effect of MB on the activity of *E. coli* ATCC25922: The bacterial suspension with 5 ml OD _600_ as 0.6–0.8 (LB broth as blank control) was taken and centrifuged at 4,000 rpm for 15 min. After the supernatant was removed, the cells were redistributed in four different concentrations (0.1, 0.2, 0.3, and 0.4 mM) of MB solution. Under the condition of strictly avoiding light, the plate colony count was carried out after being exposed to 150 rmp at 37°C for 10 min.

Electrochemical drug sensitivity test: The respiratory activity value %RA was used as an indicator of bacterial resistance by electrochemical method. The following equation has been used for calculation:

$$\%RA=\frac{\left|\text{I}0-\text{I}+\text{drug}\right|}{\left|\text{I}0-\text{I}-\text{drug}\right|}\times 100,$$

where %RA is respiratory activity; I_0_ is the current value of 0.2 mM MB; and I_-drug_ is the current value in the absence of the antibiotics. I_+drug_ is the current value in the presence of the antibiotics. A higher %RA value reflects a higher respiratory activity of bacteria, suggesting the antibiotics have little effect on bacteria.

## Results and Discussion

In order to obtain the maximum electrical signal, 0.1 mM methylene blue was scanned with graphene ink–modified gold electrode (G-Au) and graphene ink–modified glassy carbon electrode (G-GCE), respectively. It can be seen from Figure 1A that the redox electric signal of methylene blue on the G-GCE is significantly greater than that on the G-Au, which may be due to the faster electron conduction velocity of methylene blue on the carbon material than on the G-Au. Therefore, we choose the G-GCE as the working electrode of the follow-up experiment. In order to explore the relationship between MB concentration and electrochemical response signal, CV scanning was performed on 5 different concentrations of MB. As shown in Figure 1B, there is a good linear relationship between MB concentration and the peak current of CV, and the current response signal increases with the increase of MB concentration.

**FIGURE 1:** **(A)** CV of 0.1 mM methylene blue on G–Au and G–GCE. **(B)** CV curve of different concentration of MB.

As a photosensitizer, MB can damage DNA and protein of *E. coli*. In order to ensure the activity of *E. coli* ATCC25922, the plate colony count of 0.1, 0.2, 0.3, and 0.4 mM MB and 10^8^ CFU/mL *E coli* was studied. Results as shown in Table 2, the inhibitory effect of MB on *E. coli* ATCC25922 was not particularly obvious when the concentration of MB was 0.1–0.4 mM. However, with the increase of MB concentration, the colony number of 10^5^ dilution degree decreased. Therefore, the higher the concentration of MB, the greater the electrochemical signal. Finally, 0.2 mM was used as the working concentration of MB *in vivo* interaction with *E. coli* ATCC25922.

**TABLE 2:** Plate colony count of *E.coli* ATCC 25922 was determined after the interaction of MB.

Concentration of MB (mM)	10^5^	10^6^	10^7^
0	44.32	10.62	7.71
0.1	43.22	8.27	2.23
0.2	41.22	7.32	1.66
0.3	37.20	6.55	0.21
0.4	32.26	3.67	0.00

In order to explore the change of electrochemical signal of MB in *E. coli in vivo*, *E. coli* ATCC25922 was mixed with 0.2 mM MB for 7 min, and then the CV was scanned immediately. As shown in Figure 2, compared with the blank, *E. coli* ATCC25922 showed a significant decrease in the electrical signal and blue fading in the test solution. It was found that the reduction peak current of CV decreased by 35.7%, and the oxidation peak current decreased by 44.6%. This phenomenon is similar to that of Besant et al. (Besant et al., 2015) after mixing *E. coli* and azurol for a period of time. The fading of blue in the test solution is due to the reduction of blue MB to colorless L-MB by aerobic respiration of *E. coli* ATCC25922. The decrease of electrical signal after adding *E. coli* ATCC25922 is due to the fact that MB, as a redox shuttle, mediates the respiratory chain of bacteria and obtains electrons to be reduced during aerobic respiration. This results in a decrease in the concentration of the oxidized MB that can be detected in the solution, resulting in a decrease in the current value.

**FIGURE 2:** CV curve of MB in the presence and absence of *b*.

In order to explore the interaction between oxygen and MB and bacteria, the methylene blue solution with and without bacteria was deoxidized for 7 min, and the CV results are shown in Figure 3. In order to explore the interaction between oxygen and MB and bacteria, the MB solution with and without bacteria was deoxidized for 7 min, and the CV results are shown in Figure 3. It can be seen from CV that the current is lower than that without adding *E. coli* ATCC25922, no matter whether or not deoxidizing. This is due to the respiration of *E. coli*, which reduces a part of MB in the solution, resulting in the decrease of MB concentration and current. It should be noted that the current decreased more after the addition of *E. coli* with the deoxidization, which indicated that the removal of dissolved oxygen accelerated the reduction of MB by *E. coli*. The CV diagram shows that when the potential is −0.5 V, the current of adding bacteria without deoxidizing is the same as that without adding bacteria, indicating that there is no dissolved oxygen in the solution even though there is no deoxidization after adding bacteria. This is due to the respiration of living *E. coli*, which consumes oxygen in the solution. Therefore, the respiration of *E. coli* still preferentially consumes oxygen and then reduces MB in the presence of oxygen in the solution. The reduction of MB by *E. coli* can be accelerated by removing dissolved oxygen from the solution.

**FIGURE 3:** Effect of dissolved oxygen on CV signal of MB in the presence of *E. coli* ATCC25922.

In order to explore the relationship between the action time and the electrical signal, the CV diagram of *E. coli* ATCC25922 mixed with 0.2 mM MB for different time was scanned, and the results are shown in Figure 4. The figure represents the reduction of MB by *E. coli* ATCC25922. It can be seen from Figure 4 that the current remains basically unchanged in the first 0–4 min. Then, the current increased rapidly in 4–8 min and reached a stable level in 8–12 min. This shows that in the first 4 min, the oxygen in the solution has not been completely consumed. The reduction of MB by *E. coli* ATCC25922 is a slow process. At 4–8 min, the effect of oxygen was reduced, and MB was rapidly reduced by bacterial respiration. During the 8–12 min, all MB in the solution was reduced. In the experiment, it can also be observed by naked eyes that the test solution gradually changes from dark blue to colorless.

**FIGURE 4:** Current overtime for *E. coli* ATCC 25922 interacting with MB for different periods.

In order to explore the relationship between different concentrations of *E. coli* ATCC25922 and MB electrical signals, CV of different concentrations of *E. coli* ATCC25922 and 0.2 mM MB were scanned. It can be seen from Figure 5A that CV oxidation peak and reduction peak are inversely proportional to the concentration of *E. coli* ATCC25922. The correlation curve between CV reduction peak current and the concentration of *E. coli* ATCC25922 was obtained by linear fitting, and the curve is shown in Figure 5B. The regression equation was established as follows: Y = 0.266x-3.566 (*R* ^2^ = 0.9956).

**FIGURE 5:** **(A)** CV curve of MB in the presence of different concentrations of *E. coli* ATCC 25922. **(B)** Plots of peak currents vs. the concentration of *E. coli* ATCC 25922.

In order to explore the appropriate concentration of antibiotics for electrochemical drug sensitivity test, CV was used to study the change of %RA value of 0.25, 0.5, 1, and 2 g/L gentamicin with *E. coli* 25,922 and E3 for 1 h. The results are shown in Figure 6. It can be seen from the figure that the %RA value of sensitive strain ATCC25922 is basically kept below 60 within the test range of gentamicin concentration, while the %RA value of drug-resistant strain E3 is about 90 when gentamicin concentration is 0.25 and 0.5 g/L. When the concentration of gentamicin increased, although %RA began to decrease, it was still higher than that of sensitive strain ATCC25922. In order to make the electrochemical method accurately detect the difference between sensitive strains and drug-resistant strains, so as not to inhibit the respiratory activity of drug-resistant strains, 0.5 g/L was selected as the concentration of electrochemical drug sensitivity test.

**FIGURE 6:** %RA change of *E. coli* ATCC 25922 and E3 toward gentamicin.

We used electrochemical techniques to detect ciprofloxacin, gentamicin, and ampicillin in E1–E4. As shown in Figure 7, the %RA value of antibiotic resistant bacteria is almost 100. In contrast, the %RA values of bacteria sensitive to antibiotics were less than 75. When the %RA measured by electrochemical method is less than 75, it can be preliminarily determined that the bacteria are sensitive to the antibiotic. When 75<%RA<100 determined by electrochemical method, the antibiotic resistance of bacteria can be preliminarily determined.

**FIGURE 7:** %RA changes of E1–E4 toward ciprofloxacin, gentamicin, and ampicillin.

## Conclusion

In this work, CV was used to study the electrochemical characteristics of MB in the presence of *E. coli* ATCC25922. We constructed the correlation curve between the CV peak current and the concentration of *E. coli* ATCC25922. It provides a theoretical basis for electrochemical detection of bacteria. At the same time, we explored the electrochemical detection of foodborne *E. coli* drug sensitivity. The sensitivity of four *E. coli* isolates to three antibiotics was tested by the electrochemical drug sensitivity test. The results showed that bacteria were considered to be resistant to antibiotics when the standard of drug sensitivity was 75<%RA<100.

## Data Availability

The original contributions presented in the study are included in the article/Supplementary Material, further inquiries can be directed to the corresponding author.
